# Co-relation Between Calcium-Phosphorus Product and Hypertension in End-Stage Renal Disease Patients

**DOI:** 10.7759/cureus.18885

**Published:** 2021-10-19

**Authors:** Faiza Anser, Murtaza Dhrolia, Kiran Nasir, Ruqaya Qureshi, Aasim Ahmad

**Affiliations:** 1 Nephrology, The Kidney Centre Hospital, Karachi, PAK

**Keywords:** blood pressure, chronic kidney disease, hemodialysis, hypertension, calcium-phosphorus product

## Abstract

Objective

In our study, we evaluated the relation between calcium-phosphorus (Ca-P) product and various measurements of pre and post-dialysis blood pressure (BP) in hemodialysis (HD) patients.

Methods

This is a prospective, observational, cross-sectional study in which patients undergoing maintenance HD for > six months were enrolled through non-probability consecutive sampling during a six-month period from October 2020 to March 2021. Linear regression analysis was done to study the effect of the Ca-P product for each parameter of BP and regression coefficients were acquired.

Results

There was a total of 111 patients in our study, of which 59 (53.2%) were male. The mean age was 50.1± 14.4. The most common comorbid was hypertension (98.2%). The mean HD vintage of patients was 5.7 ± 5.8 years. On linear regression analysis, the Ca-P product was strongly correlated with pre-HD diastolic BP (DBP) (0.7) and post-HD mean arterial pressure (MAP) (0.7) while a moderate correlation was present with pre (0.59) and post (0.64) HD systolic BP (SBP), post-HD diastolic BP (0.68), and pre-HD MAP (0.68). On the other hand, the Ca-P product was not correlated with pre and post-HD pulse pressure (0.06 and 0.1, respectively). When the independent effect of serum calcium (Ca), phosphorus (P), and parathyroid hormone on BP was studied, P had a significant correlation with pre and post-HD SBP, DBP, and MAP.

Conclusion

Our study demonstrates a significant association of the Ca-P product and an independent high P level with pre and post-dialysis SBP, DBP, and MAP while no association was found with pulse pressure.

## Introduction

Hypertension (HTN) is a major risk factor for cardiovascular [1] and renal disease [2] while chronic kidney disease (CKD) is the most common cause of secondary hypertension. Therefore, HTN is common in CKD, with a prevalence of 59.9% in stage III while it reaches as high as 84.1% in end-stage renal disease (ESRD) [3]. After initiating hemodialysis (HD), the prevalence of HTN decreases temporarily and then again increases in chronic HD patients (70-80%) [4].

The etiology of HTN in HD is multifactorial. Sodium and volume excess are considered the major reason for HTN in HD patients; however, other mechanisms, such as arterial stiffness, activation of the renin-angiotensin-aldosterone, sympathetic nervous systems, endothelial dysfunction, sleep apnea, and the use of erythropoietin-stimulating agents, may also be involved.

Studies have also shown the association between parathyroid hormone (PTH) [5], plasma calcium (Ca) [5-6], and phosphorus (P) levels [6-7] with blood pressure (BP) in HD. While the P load has been reported to have an effect on endothelial dysfunction by increasing the production of reactive oxygen species and decreasing nitric oxide production via inhibitory phosphorylation of endothelial nitric oxide synthase [8]. Mineral metabolism disorders have also been linked to calcification of vessels with resultant arterial stiffness [9-11] and hypertension in dialysis.

Arterial stiffness secondary to arterial calcification is associated with raised systolic blood pressure (SBP) [12] and mean arterial pressure (MAP) [13], decreases diastolic blood pressure (DBP) [12], and wide pulse pressure (PP) [12] in different studies and contribute a major role to the high cardio­vascular morbidity and mortality in ESRD.

Although P and Ca homeostasis is tightly regulated in the HD population as the management of bone mineral disorders, less attention has been paid to their potential involvement in the pathogenesis of atherosclerosis or as predictors of HTN and eventually cardiovascular disease [14-16]. The removal of fluid in patients on hemodialysis leading to large differences between pre and post-blood pressure impedes a single definition of hypertension in HD patients. Therefore, different studies have shown an association of mineral metabolism disorders with varying BP measurements.

The significance of HTN and its association with morbidity in HD patients demands the identification of non-traditional correctable factors to improve clinical outcomes in patients on hemodialysis. The sparsity of data on the correlation between the calcium-phosphorus (Ca-P) product and hypertension in ESRD patients particularly from our region, developed our interest in this subject. In the current study, we evaluated the relationship between different elements associated with a bone mineral disorder with various measurements of pre and post-dialysis BP in HD patients.

## Materials and methods

This is a prospective, observational, cross-sectional study conducted in the Department of Nephrology, the Kidney Centre Postgraduate Training Institute (TKC-PGTI) after approval by the institutional ethical review committee. TKC-PGTI is a tertiary level renal care facility with a dialysis unit that accommodates 66 dialysis standards defined by European Best Practice Guidelines [17]. Nearly all long-term maintenance hemodialysis (MHD) patients are dialyzed for four hours three times a week.

A total of 111 patients of both gender, aged >18 years, undergoing maintenance hemodialysis for > six months, were enrolled after taking a written informed consent in the study through non-probability consecutive sampling during a six-month period from October 2020 to March 2021. Patients with malignancy, tuberculosis, liver cirrhosis, alcohol consumption, and gastrointestinal diseases that may have a misleading influence on calcium and phosphorus metabolism were excluded. Exclusion criteria also included patients who were non-compliant to dialysis therapy or not receiving the prescribed dialysis dose.

Serum calcium, phosphorus, albumin, and hemoglobin were routinely measured once a month while serum intact parathyroid hormone (iPTH) levels were usually measured once in three months as per our dialysis unit’s protocol. Six-month averages of serum Ca, phosphate (PO4), the Ca-P product, parathyroid hormone (PTH), albumin, and hemoglobin were calculated. Data were collected from the patient's charts, maintaining confidentiality. Pre-dialysis and post-dialysis BPs were available in patient records for each dialysis treatment. One month’s BP measurements (total of 13 readings) were averaged in each of these patients. Measurements included pre and post-dialysis systolic blood pressure (SBP), diastolic blood pressure (DBP), MAP, and PP. Age, gender, primary diagnosis, comorbids, duration of hemodialysis, average ultrafiltration during dialysis, and the number of antihypertensive medications were included in the analysis.

Statistical analysis

Data were entered and analyzed on IBM SPSS version 21, cleaning and coding of data were done before analysis. Mean ± Std and median with interquartile range (IQR) were calculated for continuous variables while frequencies with percentages were observed for categorical variables. The normality of data was checked by observing histogram, Q Q plot, box plot, and Shapiro Wilk's test. In the case of normally distributed data, Pearson correlation was computed to find any association between the calcium-phosphorus product, and different blood pressure parameters and correlation coefficient (R) were obtained. While for skewed variables, the Spearman correlation was applied. Linear regression was run to see the amount of effect of the Ca-P product on each parameter of BP and regression coefficients (R2) were acquired. A multiple linear regression analysis was performed to find adjusted regression coefficient (adjusted R2) of variables like age, gender, diabetes mellitus (DM), hemoglobin (Hb), number of antihypertensive medications, average ultrafiltration, and the Ca-P product with blood pressure. A P-value of ≤ 0.05 was considered significant.

## Results

There were 111 patients in our study, of which 59 (53.2%) were male while 52 (46.8%) were female. The mean age was 50.1 ± 14.4. The most common comorbid was hypertension, which was present in 109 (98.2%) patients, followed by diabetes mellitus 39 (35.1%) while unknown kidney disease (bilateral small shrunken kidneys) was the most prevalent primary cause of chronic kidney disease (CKD; 50 (45%)). The mean HD vintage of patients was 5.7 ± 5.8 years. Baseline characteristics of study patients are presented in Table 1.

**Table 1:** Baseline characteristics of study patients IQR: interquartile range; CKD: chronic kidney disease; HD: hemodialysis

Variable	n=111
n (%) / Mean ± Std. & Median, IQR	
Age	50.1 ± 14.1 & 51.23
Gender	
Male	59(53.2)
Female	52(46.8)
Comorbid	
Hypertension	109(98.2)
Diabetes mellitus	39(35.1)
Ischemic heart disease	6(5.4)
Asthma	2(1.8)
Thyroid disorders	3(2.7)
Renal stone disease	1(0.9)
Arthritis	1(0.9)
Hepatitis	4(3.6)
Causes of CKD	
Unknown	50(45)
Diabetic kidney disease	40(36)
Glomerulonephritis	8(7.2)
Adult polycystic kidney disease	5(4.5)
Obstructive uropathy	3(2.7)
Other	5(4.5)
HD vintage	5.7 ± 5.8 & 4,.6
Average ultrafiltration per HD	1 ± 0.7 & 2.1
Average antihypertensive medications per patient	1.5 ± 0.93 & 1.1

We found that the Ca-P product strongly correlated with pre-HD diastolic BP (0.7) and post-HD mean arterial pressure (0.7) while a moderate correlation was present with pre (0.59) and post (0.64) HD systolic BP, post-HD diastolic BP (0.68), and pre-HD mean arterial pressure (0.68). On the other hand, the Ca-P product showed no correlation with pre (0.06) and post (0.1) HD pulse pressure (Table 2).

**Table 2:** Correlation and regression coefficient of Ca-P product for blood pressure HD: hemodialysis; BP: blood pressure; MAP: mean arterial pressure; Ca-P: calcium-phosphorus

Blood Pressure parameters	Correlation coefficient	95% CI Lower-Upper	R square	P-value
Pre-HD diastolic BP	0.7	0.58-0.84	0.51	<0.001
Pre-HD systolic BP	0.59	0.52-0.81	0.43	<0.001
Pre-HD MAP	0.68	0.5-0.76	0.46	<0.001
Pre-HD pulse pressure	0.06	-0.15-0.08	0.004	0.512
Post-HD diastolic BP	0.68	0.54-0.8	0.49	<0.001
Post HD systolic BP	0.64	0.61- 0.92	0.47	<0.001
Post HD MAP	0.7	0.58- 0.83	0.53	<0.001
Post HD Pulse pressure	0.1	-0.04-0.2	0.02	0.206

The Ca-P product had a profound impact on all parameters of BP except pulse pressure. In regression analysis, we found that patient’s blood pressure HD can be significantly predicted by the Ca-P product at a p-value of <0.001. The R2 value for pre-HD DBP depicts a 51% of variability, which can be accounted for by the Ca-P product. Similarly, 43% variance in the pre-HD SBP can be explained by the product of calcium and phosphorus and 46% variation in MAP. A similar impact of the Ca-P product can be seen in the post-HD parameters of BP (Table 2).

Figure 1 shows the linear association of Ca-P product with the mean of pre and post-HD systolic, diastolic, mean arterial pressure, and PP. From the graphs, it can easily be observed that an increase in the Ca-P product causes a rise in the pre and post-HD systolic, diastolic, and mean arterial pressure. On the contrary, pre and post-PP were not linearly associated with the Ca-P product.

**Figure 1:** Linear regression between the Ca-P product and BP Ca-P: calcium-phosphorus; BP: blood pressure

We have also studied the independent effect of serum Ca, P, and iPTH on different BP readings and found that among all these, only PO4 had a significant correlation and impact on blood pressure (Table 3).

**Table 3:** Correlation and regression coefficient of serum phosphorus for blood pressure HD: hemodialysis; BP: blood pressure

Blood pressure parameters	Correlation coefficient	R square	P-value
Pre-HD diastolic BP	0.62	0.38	<0.001
Pre-HD systolic BP	0.63	0.4	<0.001
Pre-HD mean arterial pressure	0.6	0.36	<0.001
Pre-HD pulse pressure	0.05	0.002	0.603
Post-HD diastolic BP	0.6	0.36	<0.001
Post-HD systolic BP	0.62	0.39	<0.001
Post-HD mean arterial pressure	0.64	0.41	<0.001
Post-HD pulse pressure	0.19	0.035	0.048

We made eight models for the parameters of BP in multiple linear regression analysis; all models of BP had a significant impact on predicting the blood pressure of ESRD patients (p-value of analysis of variance (ANOVA) <0.001 for pre and post-systolic, diastolic BP, and MAP while p=0.027 for pre-HD pulse pressure and p=0.040 for post-HD pulse pressure). In multiple linear regression analysis, we found that the Ca-P product had a significant effect on pre and post-HD SBP, DBP, and MAP, when adjusted for age, gender, DM, Hb, the number of antihypertensive medications, and average ultrafiltration rate (p<0.001). Age was found to have a significant effect on pre-HD SBP (p=0.038) and PP (p=0.013) while gender had a significant effect on pre-HD DBP (p=0.012) and pre-HD MAP (p=0.017) when adjusted for the above-mentioned variables, including the Ca-P product. DM, Hb, the number of antihypertensive medications, and the average ultrafiltration rate had no significant effect on pre and post-BP parameters. We observed that variation in blood pressure could be better explained when we adjusted the Ca-P product with other regressors as compared to the individual effect on BP. The adjusted regression coefficients of pre and post-HD SBP, DBP, and MAP were increased in multiple linear analyses (Table 4).

**Table 4:** Multiple linear regression analysis showing variation in blood pressure Ca-P: calcium-phosphorus; HD: hemodialysis; BP: blood pressure

Blood pressure parameters	Adjusted R square	P-value
Pre-HD diastolic BP	0.53	<0.001
Pre-HD systolic BP	0.44	<0.001
Pre-HD mean arterial pressure	0.49	<0.001
Pre-HD pulse pressure	0.08	0.027
Post-HD diastolic BP	0.51	<0.001
Post-HD systolic BP	0.51	<0.001
Post-HD mean arterial pressure	0.56	<0.001
Post-HD pulse pressure	0.07	0.04

## Discussion

We observed a significant association between the Ca-P product and BP in HD patients in our study. In a regression study, the Ca-P product was positively associated with pre and post-dialysis SBP, DBP, and MAP while no association was found between the Ca-P product and pulse pressure. While in a multiple linear regression analysis, we found that the Ca-P product was the only modifiable factor among DM, Hb, the number of antihypertensive medications, and the average ultrafiltration rate that had a significant effect on pre and post-HD SBP, DBP, and MAP. When we observed the independent effect of serum Ca, PO4, and iPTH on different readings of BP, serum PO4 was found to have a positive association with pre and post-SBP, DBP, and MAP, indicating the independent effect of PO4 in the physiologic mechanism of hypertension.

Studies have shown the association between plasma calcium [6] and phosphorus [6-7] with blood pressure in HD largely attributed to vascular calcification. The development of calcification in CKD patients is strongly linked to dysregulated mineral metabolism characterized by the long-term elevation of serum phosphate levels as well as transient bouts of hypercalcemia [18]. Elevated Ca and P have a direct effect on vascular smooth muscle cells (VSMCs) that promote vascular calcification, including the stimulation of osteogenic/chondrogenic differentiation, vesicle release, apoptosis, loss of inhibitors, and extracellular matrix degradation [19].

Studies that have evaluated the correlation between the Ca-P product and BP in HD found different results in the past. A study from China found no correlation between pulse pressure and plasma PTH levels or calcium-phosphorus products [20]. A cross-sectional analysis performed to determine risk factors associated with hypertension in chronic hemodialysis patients upon enrollment into the Hemodialysis (HEMO) study found an association between serum P and higher mean and diastolic BP in HD. Another study from the USA, which studied the relationship between serum phosphate levels and blood pressure in incident hemodialysis patients, found that elevated serum phosphate was associated with higher pre-dialysis SBP and PP with a 1.77 mmHg rise in SBP for each 1 mg/dL higher phosphorous level. Ashkar ZM, in his cross-sectional study, found a significant association between the Ca-P product and pre-dialysis SBP and MAP and both pre and post-dialysis DBP [21]. No relationship was detected with PP.

Studies that found an association of pulse pressure with the Ca-P product propose that PP is directed by the association between ventricular ejection and arterial stiffness. Arterial calcifications associated with elevated Ca-P product contribute to arterial stiffness, causing an increase in PP [12,16]. Other studies that found an association of MAP with the Ca-P product explained that major MAP determinants are ventricular ejection and peripheral vascular resistance. Arterial wall hypertrophy, caused by metastatic calcifications of the arterial media or by the activation of fibroblasts, and vascular smooth muscle cells fibrosis, caused by elevated Ca and P, lead to the elevated tensile strength of arteries and result in increased peripheral resistance [22].

Our study showed a positive association of the Ca-P product and independent PO4 with MAP but no association with PP. Similar findings were found in studies from China [20] and the USA [21]. As PP is the difference between SBP and DBP, the absence of association of the Ca-P product with PP in our study likely related to the positive association with both raised SBP and DBP in our study, which suggests the predominant effect of the Ca-P product and PO4 on increasing peripheral vascular resistance in our HD patients.

Although our study is a single-center, observational, cross-sectional study, no direct causality could be established between the Ca-P product and BP measurements; however, a significant association can easily be ascertained from our study, which suggests the Ca-P product and P as important, non-traditional correctable factors and predictors of hypertension in HD patients. Extricating the complex regulatory pathways that mediate Ca and P’s effect on VSMCs will ultimately provide novel targets and therapies to limit the destructive effects of vascular calcification in CKD patients.

## Conclusions

Our study demonstrates the significant association of the Ca-P product and independent P levels with pre and post-dialysis SBP, DBP, and MAP while no association was found with pulse pressure. The Ca-P product and P are significant, non-traditional, correctable factors and predictors of hypertension in HD and need to be tightly regulated to improve clinical outcomes in patients on HD. 
